The article "Clinical Efficacy Evaluation of Psychological Nursing Intervention Combined with Drugs Treatment of Children with ADHD under Artificial Intelligence" was retracted in 2023. Reasons: unreliable results or conclusions; concerns about the data; concerns about the peer review; concerns about the citations.

# Clinical Efficacy Evaluation of Psychological Nursing Intervention Combined with Drugs Treatment of Children with ADHD under Artificial Intelligence

**DOI:** 10.1155/2022/1818693

**Published:** 2022-03-29

**Authors:** Ying Guo, Jinping Wang, Shuyan Yan, Shujie Sui

**Affiliations:** ^1^Catheter Room, The Fourth Affiliated Hospital of Harbin Medical University, Harbin 150086, China; ^2^Department of Orthopedics, The Fourth Affiliated Hospital of Harbin Medical University, Harbin 150086, China; ^3^Department of Hematology, The Fourth Affiliated Hospital of Harbin Medical University, Harbin 150086, China; ^4^School of Nursing, Harbin Medical University, Harbin 150086, China

## Abstract

ADHD in children is one of the most common neurodevelopmental disorders. It is manifested as inattention, hyperactivity, impulsiveness, and other symptoms that are inconsistent with the developmental level in different occasions, accompanied by functional impairment in social, academic, and occupational aspects. At present, the treatment for children with ADHD is mainly based on psychological nursing intervention combined with drug therapy. Therefore, the actual efficacy evaluation of this treatment regimen is very important. Neural networks are widely used in smart medical care. This work combines artificial intelligence with the evaluation of clinical treatment effects of ADHD children and designs an intelligent model based on neural networks for evaluating the clinical efficacy of psychological nursing intervention combined with drug treatment of children with ADHD. The main research is that, for the evaluation of clinical treatment effect of ADHD in children, this paper proposes a 1D Parallel Multichannel Network (1DPMN), which is a convolutional neural network. The results show that network models can extract different data features through different channels and can achieve high accuracy evaluation of clinical efficacy of ADHD in children. On the basis of the model, performance is improved through the study of Adam optimizer to speed up the model convergence, adopts batch normalization algorithm to improve stability, and uses Dropout to improve the generalization ability of the network. Aiming at the problem of too many parameters, the 1DPMN is optimized through the principle of local sparseness, and the model parameters are greatly reduced.

## 1. Introduction

Childhood ADHD, or mild brain dysfunction syndrome, is a relatively common childhood behavioral disorder syndrome. These children have normal or near-normal intelligence, hyperactivity, inattention, emotional instability, impulsive willfulness, and learning difficulties of varying degrees. ADHD can be divided into three types, namely, , inattentive, hyperactive, and impulsive [1–4].

The main harm of ADHD to children is mainly manifested in personal growth and family life. In terms of children's personal growth, because children cannot concentrate on their studies and cannot take the initiative to study, their academic performance declines. They are unable to self-control in behavior, showing disobedience and being discriminated against. As we get older, because we cannot control ourselves and are vulnerable to bad influences and temptations, we may fight, lie, and steal and even commit crimes. In terms of children's family life, due to children with ADHD, their ability to control themselves is poor, their academic performance is poor, and there will be phenomena such as weariness and truancy. Because of this, they are often criticized by teachers, making parents feel ashamed and irritable, so they often use beatings and sticks to educate their children, strictly disciplining children in their studies and adding more learning tasks to children; however, the effect is twice the result with half the effort, making children more rebellious and adopting a confrontational and hatred attitude towards parents' demands, which affects family harmony. Therefore, it is very important to achieve early recognition and early intervention to alleviate the symptoms of patients and reduce their social damage [5–8].

Childhood ADHD is considered to be a psychobehavioral disease caused by both genetic factors and environmental factors and is the result of multiple physiological, psychological, and environmental factors. (1) Physiological factors: children suffering from attention deficit hyperactivity disorder have certain familial inheritance, and various research results at home and abroad have shown this. In addition, the mother's heavy smoking and drinking during pregnancy or encountering other risks that lead to brain damage to the fetus are also a high-risk factor for children with attention deficit hyperactivity disorder. Studies have found that when children lack trace elements such as zinc and iron and the metabolism of some important amino acids in the body is out of balance, children will increase the probability of suffering from attention deficit hyperactivity disorder. (2) Psychological factors: children with ADHD are more sensitive and insecure and often use aggressive and talkative methods to cover up their inner fears and unease. If parents and teachers cannot understand their mistakes, they treat them with harsh beatings and insults. This can lead to heightened hyperactivity and even in adulthood can lead to antisocial emotions and behaviors that increase crime rates. (3) Environmental factors: in the family environment of children with ADHD, a case-control study has shown that the results show that parents' low educational level and poor family discord and intimacy are important reasons for the bad behavior of ADHD children [9–12].

Due to different research directions of ADHD children at home and abroad, the intervention methods used are also different. For children with ADHD who have obvious attention deficit and hyperactive behaviors, a common and more effective method is psychological nursing intervention combined with drug treatment [13–16]. Therefore, how to evaluate the clinical efficacy of this treatment is very important. With the development of computer technology, artificial intelligence is widely used in the field of intelligent medical care. This paper aims to design a neural network for efficient evaluation of clinical efficacy of this treatment based on artificial intelligence.

The key contribution of this study is as follows:

1. We proposed a model for the efficacy evaluation based on the 1DPMN. We used CNN for auto feature extraction from raw statistical data rather than manual feature extraction with high accuracy.
2. We optimized 1DPMN to reduce the training time by picking Adam optimizer and used batch normalization for stability of the network model.

The rest of the paper is organized as follows.  Section 2 presents the related work. The methodology applied is discussed in Section 3. In Section 4, experimental details are mentioned. Finally, Section 5 addresses the conclusion of this study.

## 2. Related Work

ADHD is one of the most common psychobehavioral disorders in children. Literature [17] proposes that the prevalence of ADHD in children worldwide is estimated to have risen to 10%. Literature [18] conducted a systematic analysis of the prevalence of ADHD among children in the United States in 2003, 2007, and 2011 and found that the prevalence of boys was 11.0%, 13.2%, and 15.1%, respectively, and the prevalence of girls was 4.4%, 5.6%, and 6.7%. Literature [19] proposed that, due to the limited awareness of ADHD and the existence of many undiagnosed cases, the prevalence of ADHD was underestimated, and the actual prevalence may far exceed this number. Literature [20] proposed that the impact of ADHD on children is reflected in academic achievement, interpersonal communication, and other aspects. Literature [21] proposed that ADHD not only affects children, but also includes the effects of comorbidities and disorders. About 66% of ADHD children have at least one comorbidity, mainly including oppositional defiant, conduct disorder, depression and anxiety, tic disorder, learning or communication disorder, sleep problems and disorders, and substance abuse. These problems and barriers can also have serious consequences for children themselves and their families. Literature [22] believes that 80% of individuals diagnosed with ADHD in childhood will continue to be between adolescence and 30 years of age. These symptoms and damage persist into adolescence and even into adulthood, and the risk of developing antisocial personality or even delinquency is 5 to 10 times that of normal children. Literature [23] believes that ADHD is a disease caused by a combination of genetic and environmental factors. Genetic studies have confirmed that ADHD is a highly hereditary polygenic genetic disease. Related genes include dopamine metabolism genes, serotonin metabolism genes, catecholamine oxygen methyl-transferase genes, and norepinephrine transporter genes. Literature [24] believes that although environmental factors have not been proven to have a causal relationship with ADHD, it is certain that environmental factors play an important role in the induction and aggravation of ADHD and the prognosis of children with ADHD. Literature [25] pointed out that the risk of ADHD in the offspring of mothers who smoked during pregnancy increased by 2.64 times, and the risk of ADHD in the offspring of mothers who drank during pregnancy increased by 1.55 times.

In [26], a CNN model LeNet-5 with a 5-layer structure was proposed, which was initially mainly used for the recognition of handwritten digits. Based on the LeNet-5 model, a large number of convolutional neural network models with different structures have also been proposed. Reference [27] proposed an AlexNet model with an eight-layer structure based on LeNet-5, which for the first time enhanced the performance of the model by using a linear rectification function and local response normalization operations during training. Therefore, AlexNet won the ImageNet Challenge with a score of 10.9% more than the second place that year, setting off a wave of deep learning since then. Reference [28] proposed the VGGNet series of models. Compared with AlexNet, which uses a 7×7 convolution kernel, VGGNet reduces model parameters by using a 3×3 small convolution kernel during the design process and increases the nonlinear expression ability of the model by stacking small-sized convolution kernels. In response to the problem that the fitting ability of CNN increases with the increase of the number of layers, ResNet is proposed in [29]. The network solves the problem of gradient disappearance and gradient explosion in the learning process of deep neural networks by means of residual learning. Reference [30] proposed the DenseNet model, which is different from the residual learning method of the ResNet model. This model avoids the risk of gradient disappearance and gradient explosion during the training process by enhancing feature transfer between layers of the network. With the continuous optimization of CNN structure and major breakthroughs in the field of pattern recognition, CNN has been gradually introduced into the medical field by scholars in recent years.

## 3. Method

### 3.1. 1D Parallel Multichannel Network

This work proposes an evaluation network 1DPMN for evaluating the clinical efficacy of psychological nursing intervention combined with drug therapy on children with ADHD. The network structure is shown in Figure 1. The input data of the network model is the original efficacy index feature. The model contains three parallel channels, and the scales of the convolution kernels used in each channel are different. The local information features of different scales of the input data are extracted through different size convolution kernels of each different channel, and these information features are highly complementary and complement each other. The tandem network structure using convolution kernels of different scales does not capture complementary informative features well. Therefore, the use of parallel multichannel convolution kernels can deeply mine the local information correlation of the internal space of the original data and reduce the semantic gap between features.

The network model consists of three parallel channels, each of which is connected by three basic unit modules. Each basic unit module includes a convolution layer and a pooling layer, and the feature information is fused in the fusion layer according to the feature information extracted from each channel. The fused information features are input into the fully connected layer, and finally the classification results are output through the Softmax layer. The specific parameter settings of the 1DPMN model are shown in Table 1.

The model contains three parallel channels, Conv1, Conv2, and Conv3, and the size and shape of the original data are expanded to 1024×1. In the first channel, the number of convolution kernels of the first convolutional layer is 64, the length and width of the convolution kernel are set to 64×1, the depth is 1, and the moving step size is 16×1. The size of the output data after the first layer of convolution is 64×64. Input the data after convolution to the first layer of pooling layer, the number of filters in the pooling layer is 64, the size of the filter length and width is 3×1, the depth is 1, the moving step size is 2×1, and the output size is 32×64.

Similarly, the convolution and pooling process of the second channel and the third channel is the same as the first channel. It can be concluded that the output data sizes of the second and third channels are 32×64 and 32×64, respectively. The output results of these three channels are passed through the fusion layer, and the features of the three channels are spliced to obtain the final feature size of 32×192. The final feature is then transported to a flattening layer, which flattens the feature to a dimension length of 6144. The output length after two fully connected layers is 512, and the final output length is 10 through the Softmax layer. The above is the specific operation process of the initial data in the entire 1DPMN model.

### 3.2. Underfitting and Overfitting

The phenomenon of underfitting is usually when the model has poor learning ability during training. Due to the insufficient learning ability of the model, it is difficult to extract the general features in the data. The performance is that the accuracy of the network model in the training set is low, the accuracy of the validation set and test set is close to the training set, and the output results have high bias characteristics, so the generalization of the model is weak. The reasons for underfitting may be caused by many factors, usually caused by the simple structure of the model, the small amount of data, the small number of model training times, the size of the batch-size, and the small amount of features of the data samples.

The phenomenon of overfitting is usually caused by the learning ability of the model being too strong. At this time, the general law of model learning is too strong. When training the model, the characteristics of a single training sample can be captured, and the model will recognize it as a general rule. This leads to the deterioration of the generalization ability of the model, which is mainly manifested in the high variance of the output results. The reasons for overfitting are also caused by various factors, generally due to the complex network model structure and too many parameters, too many model training rounds, too small training datasets, and other factors. The solution is usually to reduce the model complexity, increase the training set data, data augmentation, dropout techniques, and batch regularization, and reduce the number of model trainings, etc.

### 3.3. Adam Optimizer

In the process of deep learning model training, the internal weights and biases of the model are constantly updated iteratively, which is critical to the final performance of the model. Therefore, when training a PMCNN model, it is essentially iteratively updating its weights and biases. The optimizer plays a pivotal role in this process, and the main role of the optimizer is in the process of deep learning gradient backpropagation. It guides each parameter in the loss function to update the appropriate size in the direction of optimization, so that the updated parameters can make the loss function value continuously tend to the global minimum value. Therefore, choosing a suitable optimizer can not only speed up the model convergence speed and reduce the number of training rounds and time, but also improve the final performance of the model.

This section compares the commonly used Stochastic Gradient Descent (SGD) algorithm with the Adaptive Moment (Adam) algorithm. The SGD algorithm has lower requirements on gradients and is faster when training models on large datasets. The formula for calculating SGD is

(1) $$\begin{array}{c} \theta =\theta -\eta \nabla_{\theta }\;J\left(\theta \right),\\ v_{t}=\gamma v_{t-1}+\eta \nabla_{\theta }\;J\left(\theta \right),\\ \theta =\theta -v_{t}. \end{array}$$

In the process of model training, the learning rate is also a key factor affecting the final performance of the model. The learning rate is generally set before training the model and cannot be dynamically adjusted during the model training process. The Adam algorithm adjusts the adaptive row learning rate of each parameter by calculating the first and second moment estimates of the gradient. It is suitable for situations where the amount of data and network model parameters are large, and the update of model parameters is not affected by the scaling changes of gradients, making model training more efficient. The formula for calculating Adam is

(2) $$\begin{array}{c} {\hat{m}}_{t}=\frac{m_{t}}{\left(1-\beta_{1}^{t}\right)},\\ {\hat{v}}_{t}=\frac{v_{t}}{\left(1-\beta_{2}^{t}\right)},\\ \theta_{t}=\theta_{t-1}-\frac{\alpha {\hat{m}}_{t}}{\left(\sqrt{{\hat{v}}_{t}}+\varepsilon \right)}. \end{array}$$

### 3.4. BN Layer

Batch normalization (BN) is to solve the problem of internal covariate shift, which mainly occurs in the deep neural network training process. Because there are many layers in a deep network model, usually when the parameters of the previous layer are iteratively updated, the input data distribution of the latter layer changes. Therefore, the latter layer also needs to be continuously adjusted in the iterative process to eliminate this effect, making network training more difficult.

BN realizes the operation of preprocessing in the middle of the neural network layer; that is, the output of the previous layer is normalized and then used as an input into the next layer of the network. This can effectively prevent the gradient from disappearing and speed up network training. The BN algorithm generally performs batch normalization on the feature responses without ReLU activation. Therefore, the BN layer is placed after each convolutional layer of the network, and the processed output is used as the input of the excitation layer to achieve the effect of adjusting the partial derivative of the excitation function. The calculation of BN is as follows:

(3) $$\begin{array}{c} \mu =\frac{1}{m}\overset{m}{\underset{i=1}{\sum }}x_{i},\\ \sigma^{2}=\frac{1}{m}\overset{m}{\underset{i=1}{\sum }}{\left(x_{i}-\mu \right)}^{2},\\ {\hat{x}}_{i}=\frac{x_{i}-\mu }{\sqrt{\sigma^{2}+\varepsilon }},\\ y_{i}=\gamma {\hat{x}}_{i}+\beta , \end{array}$$

where *m* represents the size of the minibatch, *x*_*i*_ is the value in the feature map, *x*_*i*_ is a constant, and *γ* and *β* are two learnable variables. The BN layer normalizes the distribution of each layer's features by computing the mean *μ* and variance *σ*^2^ of the data in the minibatch. Moreover, the network is trained with a small batch of samples, so that the network will not generate a certain value from a given training sample, which is beneficial to improve the generalization ability of the network. Considering that the standardization operation will weaken the network's ability to express features, two learnable scaling parameters *γ* and offset parameters *β* are given to allow the network to adaptively adjust the feature distribution of the network layer.

### 3.5. Dropout

In deep learning model training, if the number of samples in the training set is too small and the model has many parameters, the network is prone to overfitting. It is mainly manifested in that the accuracy of the training set is high, while the accuracy of the test set is low; that is, the generalization ability of the model is not enough. Aiming at the above problems, this work uses the Dropout strategy to solve it. Dropout is a computationally simple and effective method that can effectively regularize neural network models and is suitable for training and testing many neural networks. The Dropout method does not have too many restrictions on the type of model or training process and is applicable to almost any model.

The idea of the Dropout method is to drop or discard nonoutput units probabilistically in the original network. This method can act on the input layer and the hidden layer, and the general probability value ranges from 0 to 0.5. In the process of model training, the mechanism of Dropout enables the neurons in the subnetwork to better transmit information and obtain more gradient change values, so it can learn more features in the dataset. During the training process, the complete neural network generates a series of subnetworks through dropout, and these subnetwork models share parameters. During testing or generalization, the final model is complete. That is, without deleting or discarding nonoutput units, the subnetworks during training share the weights into the final model, and then the final model can be regarded as the integration of these subnetworks. Therefore, the dropout method is formally an ensemble of models with shared hidden units.

### 3.6. Local Sparse Structure

In the 1DPMN model structure proposed in the previous section, the size of the convolution kernel in the same convolutional layer in each channel is the same, but the parameters of each convolution kernel are different. In the feature extraction of the original data, the use of convolution kernels of different sizes will be a new direction of neural network design. According to Hebbian theory, neurons with similar functions tend to cluster together. Using this theory, the convolution kernel in the convolution layer can be designed as a sparse structure, so that the convolution kernel with larger size can be decomposed into multiple convolution kernels with smaller size. That is, the convolution kernel with a smaller size replaces the convolution kernel with a larger convolution kernel, and each small convolution kernel is responsible for extracting a certain feature. Using this method can greatly reduce the redundant parameters of the convolutional layer and further reduce the overall parameter amount of the entire network model.  Figure 2 shows a schematic diagram of two kinds of local sparsity.

When the convolution kernel size is 3×1, two different improvement mechanisms of the local sparse mechanism guarantee the feature map size-invariant structure and dimension-changing structure. The core idea of the local sparse mechanism is to use a small convolution kernel instead of a larger convolution kernel, which is controlled by changing the size of the feature maps before and after. The other is mainly to achieve the purpose by changing the dimension size before and after the output. Increasing the 1×1 convolution is mainly to change the dimension of the feature. The dimension here mainly refers to the number of channels of the feature, not the length or width of the feature. In addition, the nonlinear excitation of the network is increased, which improves the performance of the model.

Since the size of the convolution kernel may vary, in this chapter, we mainly optimize and improve the 3×1, 5×1, and 7×1 convolution kernel layers used in the three channels of the PMDCNN model. The improved 1DPMN structure is shown in Figure 3.

## 4. Experiment Details

### 4.1. Dataset

This work uses one self-produced datasets to evaluate clinical efficacy in children with ADHD. The input features of each data sample are 10 ADHD evaluation indicators, and the specific indicator information is shown in Table 2. It should be noted that these 10 characteristic indicators were collected after psychological nursing intervention combined with drug treatment. The output for each data sample is 10 efficacy evaluation levels.

This dataset contains 2903 training samples and 1227 testing samples. The evaluation metrics are precision, recall, and F1 score in this work.

### 4.2. Evaluation for Training Progress

In convolutional neural networks and any kind of neural network, the convergence of the network is an important indicator. A network can only be used for testing tasks if it can fit effectively on the training set. Therefore, this work first evaluates the convergence of the network, and the training error and training precision of the network are shown in Figure 4.

It can be seen from the figure that with the progress of network training, the training loss gradually decreases and the training precision gradually increases. When the number of iterations exceeds 60, the loss of the network does not decrease, and the precision does not increase, which indicates that the network has converged at this time. The experimental results can ensure the reliability and robustness of the network.

### 4.3. Evaluation for Network Optimizer

As mentioned earlier, this work uses the Adam optimizer to optimize the training process of the network. To verify the effectiveness of this strategy, this work compares the network performance when using Adam optimizer and when using SGD optimizer. The experimental results are illustrated in Figure 5.

Obviously, the network gets the best performance when using the Adam optimizer. Compared to the performance when using the SGD optimizer, it can get 1.6% precision improvement, 1.4% recall improvement, and 1.2% F1 score improvement. This can prove the effectiveness and feasibility of this work using the Adam optimizer to optimize the network training process.

### 4.4. Evaluation for BN Layer

As mentioned earlier, this work uses the BN layer to constrain the distribution of feature values, thereby improving network convergence speed and accuracy. To verify the effectiveness of this strategy, this work compares the network performance when using the BN layer and when not using it. The experimental results are illustrated in Figure 6.

Obviously, the network gets the best performance when using the BN layer. Compared to the performance when not using the BN layer, it can get 1.0% precision improvement, 0.8% recall improvement, and 1.1% F1 score improvement. This can prove the effectiveness and feasibility of this work using the BN layer to optimize the network training process.

### 4.5. Evaluation for Dropout

As mentioned earlier, this work uses the Dropout strategy to deactivate certain neurons to alleviate overfitting, thereby improving network convergence speed and accuracy. To verify the effectiveness of this strategy, this work compares the network performance when using Dropout strategy and when not using Dropout strategy. The experimental results are illustrated in Figure 7.

Obviously, the network gets the best performance when using the Dropout strategy. Compared to the performance when not using the Dropout strategy, it can get 0.8% precision improvement, 0.7% recall improvement, and 1.2% F1 score improvement. This can prove the effectiveness and feasibility of this work using the Dropout strategy to optimize the network training process.

### 4.6. Evaluation on Local Sparseness

As mentioned earlier, this work uses the local sparseness (LS) to reduce network complexity, thereby improving network convergence speed and reducing training time. To verify the effectiveness of this strategy, this work compares the network training time and network parameters when using local sparseness and when not using local sparseness. The experimental results are illustrated in Table 3.

Obviously, when the local sparse strategy is used, the parameters and training time of the network are greatly optimized. This verifies the effectiveness and correctness of this strategy.

### 4.7. Comparison of Techniques

Numerous techniques were proposed in the literature and we analyzed them and made comparisons with our techniques as shown in Table 4.

## 5. Conclusion

This work mainly focuses on the clinical effect of psychological nursing intervention combined with drug therapy on children with ADHD as the research object. Aiming at the problems of traditional efficacy evaluation methods relying on expert diagnosis experience, low accuracy and low efficiency, a clinical efficacy evaluation a model for ADHD children based on deep learning theory was proposed. Through the strong automatic feature extraction ability and the strong feature learning ability of the network model, efficient efficacy evaluation can be achieved. The main research work and results of this paper are as follows. (1) Design an efficacy evaluation model based on the 1DPMN. The method uses CNN to automatically extract features from raw statistical data, instead of manual feature extraction and feature engineering, and can achieve efficacy evaluation with high accuracy. (2) The 1DPMN model is optimized. Choose the Adam optimizer to speed up model convergence and reduce training epochs and training time. The batch normalization algorithm is used to improve the stability of the network model and speed up the learning speed of the network. The use of Dropout technology improves the generalization ability of the network model and prevents overfitting. Aiming at the problem of too many parameters of the network model, the internal network structure is optimized by using the principle of local sparseness, which greatly reduces the amount of network parameters. Comprehensive and systematic experiments verify the validity and correctness of this work.

## Figures and Tables

**Figure 1:** The structure of 1DPMN.

**Figure 2:** Local sparse structures (a) and (b).

**Figure 3:** The structure of improved 1DPMN model.

**Figure 4:** Evaluation for training progress in (a) and (b).

**Figure 5:** Comparison of Adam with SGD.

**Figure 6:** Evaluation for BN layer.

**Figure 7:** Evaluation for Dropout.

**Table 1:** Design parameters of 1DPMN.

Layer	Number	Size	Stride
Conv1	64	64×1	16×1
Conv2	64	128×1	16×1
Conv3	64	256×1	16×1
Pool1	64	3×1	2×1
Pool2	64	3×1	2×1
Pool3	64	3×1	2×1
Fusion	1	-	-
Fatten	1	-	-
FC	1	1024	-
FC	1	512	-
Softmax	1	10	-

**Table 2:** Efficacy evaluation index of ADHD treatment.

Index	Detailed explanation
*i*_1_	Too much activity
*i*_2_	Excited, easily impulsive
*i*_3_	Easily disturbing other children
*i*_4_	Do things without end
*i*_5_	Often fidgets
*i*_6_	Difficulty concentrating
*i*_7_	Requirements must be met immediately
*i*_8_	Crying often, shouting loudly
*i*_9_	Emotional instability, rapid changes
*i*_10_	Unexpected behavior

**Table 3:** Evaluation on local sparseness.

Network	Parameter	Training time (h)
1DPMN	7036170	17.8
1DPMN with LS	106266	6.2

**Table 4:** Comparison of techniques.

Author and reference	Technique	Issue	Results
Susanna N. Visser et. al. [18]	Weighted analyses of 2003, 2007, and 2011 NSCH data	ADHD	Prevalence of boys was 11.0%, 13.2%, and 15.1%, respectively, and the prevalence of girls was 4.4%, 5.6%, and 6.7%
Sobanski E. et. al. [20]	Diagnostic evaluations with clinical interviews	ADHD	Prevalence of psychiatric lifetime comorbidity was 77.1%
Chen J. Y. et. al. [24]	Cross-sectional study and structural equation modelling approach	ADHD	55.6% probability of family hardiness and family support affecting family function and caregiver health directly
Our proposed method	1DPMN approach	ADHD	This method extract feature automatically and achieved high accuracy

## Data Availability

The datasets used during the current study are available from the corresponding author on reasonable request.
